The article "ECG Classification for Detecting ECG Arrhythmia Empowered with Deep Learning Approaches" was published in 2022. Journal: Comput Intell Neurosci.

# ECG Classification for Detecting ECG Arrhythmia Empowered with Deep Learning Approaches

**DOI:** 10.1155/2022/6852845

**Published:** 2022-07-31

**Authors:** Atta-ur Rahman, Rizwana Naz Asif, Kiran Sultan, Suleiman Ali Alsaif, Sagheer Abbas, Muhammad Adnan Khan, Amir Mosavi

**Affiliations:** ^1^Department of Computer Science, College of Computer Science, and Information Technology (CCSIT), Imam Abdulrahman Bin Faisal University (IAU), P.O. Box 1982, Dammam 31441, Saudi Arabia; ^2^School of Computer Science, National College of Business Administration & Economics, Lahore 54000, Pakistan; ^3^Department of CIT, The Applied College, King Abdulaziz University, Jeddah, Saudi Arabia; ^4^Department of Computer, Deanship of Preparatory Year and Supporting Studies, Imam Abdulrahman Bin Faisal University, P.O. Box 1982, Dammam 31441, Saudi Arabia; ^5^Department of Software, Gachon University, Seongnam 13120, Republic of Korea; ^6^John von Neumann Faculty of Informatics, Obuda University, Budapest 1034, Hungary; ^7^Institute of Information Engineering, Automation and Mathematics, The Slovak University of Technology in Bratislava, Bratislava 81107, Slovakia; ^8^Faculty of Civil Engineering, TU-Dresden, Dresden 01062, Germany

## Abstract

According to the World Health Organization (WHO) report, heart disease is spreading throughout the world very rapidly and the situation is becoming alarming in people aged 40 or above (Xu, 2020). Different methods and procedures are adopted to detect and diagnose heart abnormalities. Data scientists are working on finding the different methods with the required accuracy (Strodthoff et al., 2021). Electrocardiogram (ECG) is the procedure to find the heart condition in the waveform. For ages, the machine learning techniques, which are feature based, played a vital role in the medical sciences and centralized the data in cloud computing and having access throughout the world. Furthermore, deep learning or transfer learning widens the vision and introduces different transfer learning methods to ensure accuracy and time management to detect the ECG in a better way in comparison to the previous and machine learning methods. Hence, it is said that transfer learning has turned world research into more appropriate and innovative research. Here, the proposed comparison and accuracy analysis of different transfer learning methods by using ECG classification for detecting ECG Arrhythmia (CAA-TL). The CAA-TL model has the multiclassification of the ECG dataset, which has been taken from Kaggle. Some of the healthy and unhealthy datasets have been taken in real-time, augmented, and fused with the Kaggle dataset, i.e., Massachusetts Institute of Technology-Beth Israel Hospital (MIT-BIH dataset). The CAA-TL worked on the accuracy of heart problem detection by using different methods like ResNet50, AlexNet, and SqueezeNet. All three deep learning methods showed remarkable accuracy, which is improved from the previous research. The comparison of different deep learning approaches with respect to layers widens the research and gives the more clarity and accuracy and at the same time finds it time-consuming while working with multiclassification with massive dataset of ECG. The implementation of the proposed method showed an accuracy of 98.8%, 90.08%, and 91% for AlexNet, SqueezeNet, and ResNet50, respectively.

The article "ECG Classification for Detecting ECG Arrhythmia Empowered with Deep Learning Approaches" was published in 2022. Journal: Comput Intell Neurosci.

## 1. Introduction

Heart abnormalities are rising with the passage of time and people worry about the health of the entire world. Till today, ECG signals are the best procedure to detect heart abnormality and functionality. For decades, the irregular functionality of the heart has been seen [1]. A lot of heart and cancer problems are gradually increasing because of the sedentary and lethargic lifestyle [2]. A healthy heart activity can be seen with ECG and its related terminologies like P wave, QRS complex, T wave, and QT interval. The abnormality can be detected by reading these features or electrical waves with precise and accurate medical knowledge. The deep learning methods worked and observed the heart conditions that affect the heart rate [3]. Because of the improper signal, the heart rate can be slow, fast, or unforeseen. If the proper treatment will not be taken, then it leads to heart stroke and heart failure. A normal healthy person's ECG is represented by Normal Sinus Rhythm (NSR). The other condition is a chronic condition where the blood pumping is affected, and it is represented by Congestive Heart Failure (CHF). Because of the inappropriate blood circulation, the heart becomes weaker, and its functionality affects at a high rate and frequency [4, 5].

It is important to find the abnormalities in the heart and its ECG signal and to classify them [5]. The deep learning approach can best suit the problem, and having many layers of neurons of a neural network can find the method to detect the ECG signal in less time with accurate results [6]. Deep learning is already in practice to do a variety of tasks in pattern and image recognition and motivated the medical research to work in this state of the art [3–6].

The current work of the CAA-TL model is based on a transfer learning approach by using three different deep learning methods and in the previous approaches, the researcher worked on machine learning which is slow and has handcrafted features. We tried our level best to make our model novel in terms of accuracy and computational aspect. For this purpose, we have augmented images to increase the number of datasets along with different image positions.

The article "ECG Classification for Detecting ECG Arrhythmia Empowered with Deep Learning Approaches" was published in 2022. Journal: Comput Intell Neurosci.

The model worked on transfer learning which is itself an innovative approach but working with different deep learning models satisfies us which one method is better and to what extent. All these methods give the accuracy to a satisfactory level, but few classes are not trained according to our requirements. If we can work further on that and make some changes in the datasets and layers of the methods, we can get a 100% result, and for this purpose, we will try K-fold validation and other related techniques in the future, along with federated learning approach to make it reliable and secure.

The 1^st^ part is an introduction, the 2^nd^ part is a literature review, and the last is the method and results. The system architecture and performance evaluation of the proposed model justify the purpose of this paper. Finally, the conclusion part will have to evaluate the overall performance of the proposed model in light of innovative transfer learning techniques.

## 2. Literature Review

The anesthesiologist uses the ECG to get the patient's condition. A physician who has the experience still misjudges the signals sometimes. The convolutional neural network is used to classify the images to aid in anesthesia. During the research, three models, ResNet, SqueezeNet, and AlexNet, used and showed the accuracy and waveform as 0.97, 0.75, and 0.96, respectively [7].

The cardiac disorder is life-threatening and timely detection and treatment can save a life. The CNN approach can be helpful for the detection of Shockable Ventricular Cardiac Arrhythmia (SVCA). The model using the CNN approach has an average accuracy of 97.59% [8]. The machine learning approach using the manually extracted features utilizes the ECG signals. Multimodal Image Fusion (MIF) and multimodal Feature Fusion (MFF) can be used for the ECG heartbeat classification. As the input of this fusion, the ECG is converted into different images by using Gramian Angular Field (GAF), Recurrence Plot (RP), and Markov Transition Field (MTF). The experiment was done on the MIT-BIH dataset for five arrhythmia conditions and achieved the required accuracy [9].

The current methods are not considered to work at a satisfactory level. The 1-D Convolutional Neural Network (1-D CNN) is efficient, fast, and easy to use. With the 1-D CNN, the accuracy reached 91.33% for Cardiac Arrhythmic disorders and the classification time was 0,015 Seconds [10].

The researcher proposed the system of Ordinary Differential Equation (ODE) to signify the heart's dynamic forces and conditions and incorporate the ODE into a generative adversarial network to create the ECG samples [11].

The article "ECG Classification for Detecting ECG Arrhythmia Empowered with Deep Learning Approaches" was published in 2022. Journal: Comput Intell Neurosci.

The datasets of different healthy and unhealthy persons have been taken and compared to find the best accuracy and outcome. In this respect, the layers have been changed to compare the result as well [12].

The Residual Convolution Neural Network (ResNet) Attention is used for the authentication of humans by using ECG signals. The recently used methods are password, tokens, retina, etc., but towards the innovative approach, the ECG plays a vital role in the authentication. Hammad et al. proposed two models, CNN and ResNet, for human authentication. Hence, the proposed models give incredible accuracy in terms of human authentication and a broader vision in the health sciences [13].

The ECG biometric models can be trained based on the previous ECG data and get the advanced and future ECG data. The MIT-DB and ECG-ID datasets are used with two models, AlexNet and ResNet18, and gave 94.4% accuracy on ECD-ID, which promised that the ECG biometric system is good enough to identify human biometric [14].

Blood Pressure (BP) estimation can be evaluated by the ECG signals. In this regard, the machine learning approaches are applied to extract the features for the classification regression module for DBP (Diastolic Blood Pressure), Systolic Blood Pressure (SBP), and Mean Arterial Pressure (MAP). By using the training, validation, and testing evaluation, the method achieves the absolute error of 8.64 mmHg for SBP, 13.52 for MAP, and 18.20 mmHg for DBP. The experiment showed the result achieved by the method was close to BP estimation [15].

Acharya et al. proposed the diagnostic tool for Myocardial Infarction cardiovascular disease. Therefore, they proposed a novel approach for the detection of normal and abnormal ECG with noise and without noise and achieved the accuracy of 93.53% with noise and 95.22% without noise removal, respectively [16]. A voting scheme was applied amid the leads to diagnose the arrhythmia for multiple datasets. Leveraging the transfer learning SqueezeNet model for image classification, the ECG signals are converted to scalograms before going through the training process. By this, the achieved validation score is 0.214 and the full test score is 0.205, respectively [17–19].

Nitin and Sudarshan analyzed the different models of transfer learning to diagnose heart arrhythmia. Three classes, Normal Sinus Rhythm (NSR), Atrial Return Rate (ARR), and Congestive Heart failure (CHF), are used to make the Continuous Wavelet Transform (CWT) give the 2-D time-frequency of ECG signals. Three different CNN architectures like GoogleNet, AlexNet, and SqueezeNet were used, and a further transfer learning approach has done some modifications in the layers to get the accuracy of 97.8%, 97.80%, and 97.22%, respectively [20].

The article "ECG Classification for Detecting ECG Arrhythmia Empowered with Deep Learning Approaches" was published in 2022. Journal: Comput Intell Neurosci.

The blood parameters and ECG in squeezed fish can stimulate the effect of mortality, damage, and recovery. The rubber bands are tied at the head portion of the fish, which can affect the survival rate and encounter the gills nets. The blood is clotted and can pass the ECG to lead to mortality [21].

Aston et al. applied a deep learning approach to attractor images from ECG signals to detect the genetic mutation among wild-type and mutant mice. The mutation relates to the cardiac channel function and links with the ventricular arrhythmogenic risk that can be a cause of sudden death. From the waveform, they generated the attractor from ECG by using all waveform available data. To fine-tune the network, the layers have been changed in the transfer learning approach, high accuracy has been achieved, and its good practice for detecting genetic mutation from ECG signals has been proved [22].

Xu et al. interpreted the ECG disease by using CNN and RNN for detection purposes. The network used the 2 convolutional layers, ReLU activation, which was observed by bidirectional long short-term memory (biLSTM) layers. The MIT-BIH dataset was used and achieved an accuracy of 95.90% [23].

Furthermore, the automatic classification of ECG can be done by the rule-based method and deep learning network approach. The rule-based method used the time-frequency and morphological ECG features with labels and gave a validation score of 0.325 for the rule-based method and 0.426 for the deep learning method as GoogleNet [24].

Lopez et al. proposed that based on MEG activity with a randomized Convolutional network, the early stage of Alzheimer's disease can be detected [25]. Singh et al. proposed the attention-based convolutional denoising auto decoder for two different lead ECG denoising and arrhythmia classifications [26].

Ghazal et al. [27] proposed the model for detecting Alzheimer's disease detection empowered with transfer learning and trying to resolve the problem of dementia for old-aged people and get the required accuracy.

Researchers worked on a light encryption technique to secure the patient imaging data and there are a lot of problems like loss of data, data size limitations, redundancy, etc., and can be solved by using this technique and sharing it among the eHealth centers and the organizations. Furthermore, to improve the Healthcare framework, data mining techniques are used which are based on Fischer Linear discrimination and Quadratic discrimination analysis. Using these data mining techniques makes it possible to evaluate online advertisement with feature extraction and selection. The Internet of things (IoT) is playing a vital role in health science and their related fields as well and distributes the household work with productive machines with a variety of sensors and applied deep learning networks for the Internet of things applications ease the life in a variety of ways [28–31].

The article "ECG Classification for Detecting ECG Arrhythmia Empowered with Deep Learning Approaches" was published in 2022. Journal: Comput Intell Neurosci.

Heart disease was predicted by feature reduction and rule-based fuzzy classifier and performed an experiment on UCI datasets and attained an accuracy of 76.51% [32]. Furthermore, the Bio imaging-based machine learning algorithm seems to be helpful for the detection of breast cancer which is considered to have a high mortality rate throughout the world [33]. The artificial intelligent approach is widely used in colorectal cancer disease by using scaled dilation in CNN, and by using the transfer learning, the malignancy detection in lungs and colon can be cured while working with the class selective image processing [34, 35].

Shahan et al. proposed a machine learning approach to diagnose the early detection of cardiovascular disease and worked on different parameters which relate to the heart functionality as well and got a precision accuracy of 87.05% by using fuzzy logic [36].

### 2.1. Limitations of the Related Work

The previous studies have a few limitations:

- The number of images is less, and the dataset is not augmented [5, 32, 34].
- Having low accuracy [2, 6, 14, 16, 32, 36].
- Handcrafted [5, 6, 32, 34, 36].

The major contribution of this paper is listed:

- Earlier research has feature-based datasets. Here image processing and augmentation are applied to get the images of different parameters and increase the number of images as well.
- Furthermore, three different deep learning methods (AlexNet, SqueezeNet, ResNet50) were applied to check the validation of the system.
- The experiments are conducted on 16879 images, and a further 80% of images are taken for training, and 20% are taken for validation.

Table 1 shows the limitation of the previous work and its finding.

## 3. Materials and Methods

### 3.1. Dataset and Preprocessing

The dataset's multiclass ECG classification is taken from Kaggle [38]. The five different classes have the images like F (3000), N (3879), Q (2500), S (4000), and V (3500), respectively. The overall ECG images taken for training and validation are 16879. The actual number of MIT-BIH ECG images taken in the proposed CAA-TL model is different from the original, so some of the images are augmented to increase the number of images in the datasets. Then, preprocess the images to get the required dimensions of 227 × 227 according to the requirement of the transfer learning methods.  Table 2 shows the pseudocode of the proposed CAA-TL model to show the step-by-step method.

The article "ECG Classification for Detecting ECG Arrhythmia Empowered with Deep Learning Approaches" was published in 2022. Journal: Comput Intell Neurosci.

The proposed CAA-TL model showed the accuracy against each deep learning approach, but before getting the accuracy, the transfer learning methods are applied and tuned in some layers required to get the more accurate result of the proposed CAA-TL model.  Figure 1 shows the proposed architecture of CAA-TL, and it is comprised of Data acquisition, Preprocess Layer, Training layer, Validation layer, Performance, prediction, and storage layer.

There are a few steps where the ECG data is collected from Kaggle as a Data Acquisition layer. Then its preprocessed, transfer learning approach was employed to images and trained. Further, the validation process is applied to import the trained model to real-time acquisition. The training and validation worked in the ratio of 80 : 20 and got the confusion matrix against that. Three deep learning approaches, AlexNet, SqueezeNet, and ResNet50, are used and applied to the transfer learning approach by employing some layers and creating new layers of different deep learning methods.  Table 3 shows the actual picture of 80%–20% for training and validation for the entire augmented dataset.

According to the requirement in the proposed CAA-TL model, we updated the last 3 layers named: fully connected, SoftMax, and classification layer of the AlexNet model.  Figure 2 shows the validation accuracy and miss rate, and the confusion matrix is drawn against the multiclasses and gets 98.38% accuracy for the AlexNet transfer learning approach.  Table 4 shows the matrix values of training and validation of the proposed CAA-TL model of AlexNet.

Furthermore, Figure 3 shows the validation accuracy and miss rate for SqueezeNet, and the confusion matrix is drawn against the multiclassification and achieved 90.08% accuracy overall. SqueezeNet transfer learning approach showed the accuracy for the 3 classes Q, S, V, and F is 100%, 100%, and 99.9%, 43.5% but unable to detect the Class N and find NaN% as failed case, and it is declared that this transfer learning method is not able to train it, but for the other three classes, its performance is outstanding. But N class still shows 77.02% with a miss rate of 22.98% for training and accuracy 83.95% and a miss rate of 16.04% is for validation.  Table 5 shows the confusion matrix values of the proposed CAA-TL model using SqueezNet during the training and validation phases.

Furthermore, Figure 4 shows the validation accuracy and miss rate, and the confusion matrix is drawn against the multiclassification and achieved 91% accuracy overall for ResNet50.  Table 6 shows the accuracy for the 3 classes Q, S, V, and F is 100%, 100%, and 99.9%, 43.6% but unable to detect the Class N and found NaN% as failed case, and this transfer learning method is not able to train it. But still shows 77.19% with a miss rate of 22.81% and validation accuracy is 79.25% and miss rate is 20.75%.

The article "ECG Classification for Detecting ECG Arrhythmia Empowered with Deep Learning Approaches" was published in 2022. Journal: Comput Intell Neurosci.

It is concluded that the AlexNet can train and validate all the classes and achieve the best result as compared to the other two transfer learning approaches (SqueezeNet and ResNet50). But the improvement in the dataset of the N class can lead to the best result for the other two approaches as well.

## 4. Simulation and Results

A Matrix involves accuracy, miss rate, specificity, sensitivity, false negative, precision, and precision to assess the performance of different deep learning methods (AlexNet, SqueezeNet, and ResNet50) and applied the transfer learning approach in terms of changing some layers to get the required accuracy and result. MATLAB 2021a is used for simulation with high performing PC processor of 11th Gen Intel(R) Core (TM) i5-1135G7 @ 2.40 GHz, RAM 8.00 GB, and hard drive 1 TB. The performance of the proposed CAA-TL model can be calculated by the following formulas [39]:

(1) $$\begin{array}{c} \text{Accuracy}=\frac{M_{ri}/I_{ri}+M_{rk}/I_{rk}}{M_{ri}/I_{ri}+\sum_{j=1}^{n}M_{\left(rj,j\neq i\right)}/I_{rj}+M_{rk}/I_{rk}+\sum_{l=1}^{n}M_{\left(rl,l\;\neq k\right)}/I_{rk}\;}\;\text{where }i,j,k,l=1,2,3,\ldots ,n, \end{array}$$

(2) $$\begin{array}{c} \text{MissRate}=\frac{\sum_{l=1}^{n}M_{rl,l\neq k}/I_{rk}}{\sum_{l=1}^{n}M_{rl,l\neq k}/I_{rk}+M_{ri}/I_{ri}}\;\text{where}i,k,l=1,2,3,\ldots ,n, \end{array}$$

(3) $$\begin{array}{c} \frac{\text{TruePositiveRate}}{\text{Recall}}=\frac{M_{ri}/I_{ri}}{M_{ri}/I_{ri}+\sum_{l=1}^{n}M_{rl,l\neq k}/I_{rk}\;}\;\text{where}i,k,l=1,2,3,\ldots ,n, \end{array}$$

(4) $$\begin{array}{c} \frac{\text{TrueNegativeRate}}{\text{Sensitivity}}=\frac{\;M_{rk}/I_{rk}}{\;M_{rk}/I_{rk}+\sum_{j=1}^{n}M_{rj,j\neq 1}/I_{rj}}\;\text{where}j,k=1,2,3,\ldots \ldots ,n, \end{array}$$

(5) $$\begin{array}{c} \text{Precision}=\frac{M_{ri}/I_{ri}}{M_{ri}/I_{ri}\;+\;\sum_{j=1}^{n}M_{\left(rj,j\neq 1\right)}/I_{rj}}\;\text{where}i,j=1,2,3,\ldots \ldots ,n, \end{array}$$

(6) $$\begin{array}{c} \text{FalseOmissionRate}=\frac{\sum_{l=1}^{n}M_{rl,l\neq k}\;/\;I_{rk}}{\sum_{l=1}^{n}M_{\left(rl,l\neq k\right)}/I_{rk}+M_{rk}/I_{rk}}\;\text{where}k,l=1,2,3,\ldots \ldots ,n, \end{array}$$

(7) $$\begin{array}{c} \text{FalseDiscoveryRate}=\frac{\sum_{j=1}^{n}M_{rj,j\neq i}\;/I_{rj}}{M_{ri}/I_{ri}+\sum_{j=1}^{n}M_{\left(rj,j\neq i\right)}/I_{rk}j}\;\text{where}i,j=1,2,3,\ldots ..\ldots ,n, \end{array}$$

(8) $$\begin{array}{c} F0.5\text{score}=1.25\text{xPrecisionx}\frac{\text{Recall}}{0.25\text{xPrecision}+\text{Recall}}, \end{array}$$

(9) $$\begin{array}{c} F1\text{Score}=2\text{xPrecisionx}\frac{\text{Recall}}{\text{Precision}+\text{Recall}}. \end{array}$$

Table 7 represents the simulation result of all ECG classes (F, S, Q & N) using different transfer learning approaches named as AlexNet. SqueezNet & ResNet50 Hence, the AlexNet can fit best to train and validate the ECG multiclassification and get the maximum accuracy as compared to the other transfer learning approaches (SqueezeNet, and ResNet50).

The article "ECG Classification for Detecting ECG Arrhythmia Empowered with Deep Learning Approaches" was published in 2022. Journal: Comput Intell Neurosci.

The accuracy rate is good for other transfer learning approaches for a few classes, not all. Comparatively SqueezeNet and ResNet50, AlexNet can train and validate well all the classes of ECG Arrhythmia and give the accuracy against training set and validation dataset. But for SqueezeNet and ResNet50 S, some of the classes show NaN in training and validation. Here, for all the transfer learning approaches, the dataset (images) with a resolution of 270 × 270 with multiclassification. While during the training set and validation set, a few classes for ResNet50 and SqueezeNet showed the NaN still worked with different learning rates 1*e* − 1, 1*e* − 5, 1*e* − 10, 1*e* − 20, and solver side but still got the same condition as NaN. Then we also changed the layer parameters, but the results did not change. This simulation proved that at the moment, for all classes, the AlexNet is better as compared to others but changing the datasets and solver like Adam and changing the weights and the bias of different layers with the minimum values can change the accuracy of the NaN for particular classes. At the same time, the SqueezeNet and ResNet50 networks have outstanding accuracy for the classes V, S, and Q and need to work on the N and F classes by improving their dataset.  Table 8 shows the percentage Accuracy of different transfer learning approaches for the proposed CAA-TL model and discovered that all three different transfer learning approaches performed well.

### 4.1. Comparative Analysis

It has been proved that the transfer learning approach gives the fastest and most reliable result as compared to machine learning and amid a comparison of three different transfer methods, AlexNet is the most excellent method for the proposed CAA-TL model.

Table 9 shows the comparison of previous studies with the proposed CAA-TL model and proposed findings. N.Strodthoff et al. [2] used the ResNet and Inception method by using the dataset PTB-XL and the predicted accuracy is 89.8%. Wasimuddin et al. [5] used the ECG-ID dataset and applied the CAD and machine learning with an accuracy rate of 98.5%, but it is taking more time as it is handcrafted. T. Vijayakumar et al. [6] used feature extraction to remove the noise and make the system noise-free to prove the higher accuracy which is 94.5%. P.Y. Hsu et al. [14] used the transfer learning approach AlexNet and ResNet, and its predicted accuracy is 94.4% by using the dataset MIT-BIH. U.R. Acharya et al. [16] used PTB-DB and worked on CNN layers and showed an accuracy of 93.5% with noise and 95.22% without noise. G. Gaddam et al. [37] used AlexNet with predicted accuracy of 95.6%. Reddy and Khare [32] used the UCI dataset for the problem and applied a rule-based fuzzy classifier and feature reduction with an accuracy of 76.51%. Poudel et al. used the KVASIR dataset and used a method of CAD and machine learning with an F1-Score of 0.88.

The article "ECG Classification for Detecting ECG Arrhythmia Empowered with Deep Learning Approaches" was published in 2022. Journal: Comput Intell Neurosci.

## 5. Conclusions

The algorithm, ECG devices, data set, and environmental and economic considerations all have a significant role in determining the effectiveness of ECG analysis in a variety of ways. The most important thing in heart arrhythmia is to diagnose it early on to save a life, and the ECG is the greatest way to examine how the heart signals are working and early detection can lead to early treatment and can save one's life. In this work, three different fundamentally unique deep learning models were altered and considered to assess the multiclass ECG signal arrhythmia. Initially, the dataset MIT-BIH has taken from Kaggle and augmented to increase the number of images and change its parameters and positioning in a different direction. The proposed CAA-TL model showed incredible accuracy for three different deep learning models and applying transfer learning techniques by changing the layers can lead to progress in detecting and diagnosing the multiclassification of ECG. AlexNet so far proved the awesome result in terms of accuracy as compared to the other two methods (SqueezeNet and ResNet50), but still, their three classes showed the remarkable result of 100% and working with other classes in the future, the result can be more accurate and considerable in ECG arrhythmia. It is proven that all the deep learning methods are great compared to machine learning and old techniques and approaches.

In the previous research, the researcher used one or two or sometimes different transfer learning approaches, and on the same time researcher worked on feature-based methods which are handcrafted which is slow and time-consuming, but here, we have used three transfer learning approaches and found their accuracy for the ECG Arrhythmia which made our research innovative and applied augmentation on datasets as well.

The article "ECG Classification for Detecting ECG Arrhythmia Empowered with Deep Learning Approaches" was published in 2022. Journal: Comput Intell Neurosci.

There are a few future things that should be considered to get more accurate results.

Firstly, work on the dataset and improve the images of the classes, which shows less accuracy as all the parameters in respect of algorithm and architecture are checked but still getting NaN for specific classes for two deep learning approaches. More refinement can be seen by working on the dataset. Secondly, the computation complexity of this model is significant, and the validation process takes a lot of time while working for three different models to train and validate. Furthermore, we can improve the computational speed by using the GPU or AWS cloud computing service instead of using CPU and apply the innovative approach of federated deep learning to the proposed model in the future to make it more reliable and consistent in the health sciences, and the significant approach of federated learning is to centralize the system or organization's data appropriately without sharing the organization's data, which is a good step toward revolution and security. Federated deep learning can introduce the learning paradigm where the methods are trained and distributed among different networks. Nowadays, many devices and systems are interconnected and the complexity of sharing and keeping their privacy is the main problem that can be solved by federated learning. Finally, the K fold Cross-validation method is extensively used in machine learning and can be utilized to acquire and compare results for the suggested model.

## Figures and Tables

**Figure 1:** Proposed architecture of CAA-TL.

**Figure 2:** Proposed CAA-TL (AlexNet) validation accuracy and loss graph.

**Figure 3:** Validation accuracy and loss of proposed CAA-TL (SqueezeNet).

**Figure 4:** Validation accuracy and loss of proposed CAA-TL(ResNet50).

**Table 1:** Limitations of previous work.

Studies	Dataset	Method	Findings	Limitations

Strodthoff et al. [2]	PTB -XL	ResNet and inception	Predicted accuracy 89.8%	-No data augmentation
				-Less accurate

Wasimuddin et al. [5]	ECG-ID	CAD and machine learning	Predicted accuracy 98.5%	-Handcrafted
				-Small dataset

Elgendi and Menon [6]	SRAD	Database supervised ML algorithms	Predicted accuracy 75.02%	-No data augmentation
				-Handcrafted

Hsu et al. [14]	MIT-DB	AlexNet and ResNet	Predicted accuracy 94.4%	-No data augmentation

Acharya et al. [16]	PTB DB	CNN layers	Accuracy 93.5% with noise and 95.22% without noise	-Less accurate
				-Less number of classes

Gaddam et al. [37]	MIT-DB	Alex net	Predicted accuracy 95.6%	-Less accurate
				-No data augmentation

Reddy and khare [32]	UCI dataset	Rule-based fuzzy classifier and feature reduction	Predicted accuracy 76.51%	-Handcrafted
				-No augmentation
				-Less accurate

Poudel et al. [34]	KVASIR dataset	CAD and machine learning	F1-score of 0.88	-Handcrafted
				-No augmentation
				-Less number of classes

Siddique et al. [39]	Private	Fuzzy inference system, deep extreme machine learning, and ANN	87.05%, 92.45%, and 89.4%	-Handcrafted
				-No augmentation
				-Less accurate

The article "ECG Classification for Detecting ECG Arrhythmia Empowered with Deep Learning Approaches" was published in 2022. Journal: Comput Intell Neurosci.

**Table 2:** Pseudocode of the proposed CAA-TL model.

1	Start
2	Input ECG data from kaggle
3	Augmented data
4	ECG preprocess data
5	Load data & pre-trained (transfer learning) model
6	Trained model using transfer learning (AlexNet, SqueezeNet, and ResNet50) for ECG classification
7	Validation phase for ECG classification for unknown images
8	Compute the performance and accuracy of the proposed model
9	Stop

**Table 3:** Training and validation ratio of proposed CAA-TL model

Proposed CAA-TL model training and validation (80%–20%)			
AlexNet, SqueezeNet, ResNet50			
Classes	Actual number of images	Training (80%)	Validation (20%)

F	3000	2400	600
N	3879	3103	776
Q	2500	2000	500
S	4000	3200	800
V	3500	2800	700
Total	16879	13503	3370

**Table 4:** Confusion matrix of CAA-TL model (training & validation).

Images	Confusion matrix					Confusion matrix				
	CAA-TL model (AlexNet)					CAA-TL model (AlexNet)				
	80% samples for training					20% samples for validation				

F	2277	4	15	87	111	547	3	7	28	7
N	6	3090	4	2	14	1	769	2	0	10
Q	7	0	1916	48	3	1	0	473	15	0
S	86	1	49	3036	40	20	1	13	748	0
V	124	8	16	27	2632	31	3	5	9	1047

**Table 5:** Confusion matrix of CAA-TL model (training & validation).

Images	Confusion matrix					Confusion matrix				
	CAA-TL model (squeezeNet)					CAA-TL model (squeezeNet)				
	80% samples for training					20% samples for validation				

F	2500	3103	0	0	0	599	776	1	0	0
N	0	0	0	0	0	0	0	0	0	0
Q	0	0	2000	0	0	0	0	499	0	0
S	0	0	0	3200	0	0	0	0	800	1064
V	0	0	0	0	2800	1	0	0	0	0

**Table 6:** Accuracy and loss rate of ResNet50.

Dataset	Confusion matrix					Confusion matrix				
	CAA-TL model (squeezeNet)					CAA-TL model (squeezeNet)				
	80% samples for training					20% samples for validation				

F	2500	3103	0	0	0	600	776	0	0	0
N	0	0	0	0	0	0	0	0	0	0
Q	0	0	2000	0	0	0	0	500	0	0
S	0	0	0	3200	0	0	0	0	800	1064
V	0	0	0	0	2800	0	0	0	0	0

**Table 7:** Simulation result of proposed CAA-TL model.

	AlexNet		SqueezeNet		ResNet50	
Image dimensions	227 × 227		227 × 227		227 × 227	
Layers	25		68		177	

For F	Training	Validation	Training	Validation	Training	Validation
Accuracy	97.38%	76.67%	77.19%	79.20%	77.19%	79.25%
Miss classification rate	2.62%	3.23%	22.81%	20.80%	22.81%	20.75%
Sensitivity	92.40%	91.30%	44.62%	43.53%	44.62%	43.60%
Specificity	98.32%	97.34%	100%	58.21%	100%	100%
Precision	91.17%	91.08%	100%	99.83%	100%	100%
FPR	0.02%	0.03%	0%	0.99%	0%	0%
FNR	0.08%	0.09%	0.55%	0.56%	0.55%	0%

For S	Training	Validation	Training	Validation	Training	Validation
Accuracy	97.70%	97.50%	100%	71.55%	100%	71.55%
Miss classification rate	2.30%	2.5%	0%	28.45%	0%	30.66%
Sensitivity	95.66%	94.52%	100%	42.92%	100%	42.92%
Specificity	98.24%	98.42%	100%	100%	100%	100%
Precision	93.5%	94.88%	100%	100%	100%	100%
FPR	0.02%	0.02%	0%	0%	0%	0%
FNR	0.04%	0.06%	0%	0.57%	0%	0%

For Q	Training	Validation	Training	Validation	Training	Validation
Accuracy	98.85%	98.96%	100%	99.97%	100%	100%
Miss classification rate	1.15%	1.04%	0%	0.027%	0%	0%
Sensitivity	96.73%	97.61%	100%	100%	100%	100%
Specificity	99.17%	99.28%	100%	99.97%	100%	100%
Precision	94.6%	95.8%	100%	99.8%	100%	100%
FPR	0.008%	0.007%	0%	0.0003%	0%	0%
FNR	0.03%	0.02%	0%	0%	0%	0%

For N	Training	Validation	Training	Validation	Training	Validation
Accuracy	99.47%	99.74%	77.19%	83.96%	77.19%	79.25%
Miss classification rate	0.53%	0.29%	22.81%	16.04%	22.81%	20.75%
Sensitivity	98.34%	99.17%	0%	0%	0%	0%
Specificity	99.76%	99.87%	100%	83.96%	100%	79.25%
Precision	99.10%	99.58%	0%	0%	0%	0%
FPR	0.002%	0.001%	0%	0.16%	0%	0.21%
FNR	0.017%	0.008%	1%	1%	1%	1%

For V	Training	Validation	Training	Validation	Training	Validation
Accuracy	99.26%	97.48%	100%	71.52%	100%	71.55%
Miss classification rate	1.74%	2.52%	0%	28.48%	0%	28.45%
Sensitivity	95.62%	93.77%	100%	0%	100%	0%
Specificity	99.36%	98.44%	100%	71.54%	100%	71.55%
Precision	98.40%	94%	100%	0%	100%	0%
FPR	0.006%	0.02%	0%	0.28%	0%	0.28%
FNR	0.04%	0.06%	0%	1%	1%	1%

The article "ECG Classification for Detecting ECG Arrhythmia Empowered with Deep Learning Approaches" was published in 2022. Journal: Comput Intell Neurosci.

**Table 8:** Percentage accuracy of transfer learning approaches for proposed CAA-TL model.

Percentage accuracy of different classes of CAA-TL model						
Classes	AlexNet		SqueezeNet		ResNet50	
	TR	VL	TR	VL	TR	VL

V	99.26%	97.48%	100%	71.52%	100%	71.52%
S	97.70%	97.50%	100%	71.55%	100%	71.52%
Q	98.85%	98.96%	100%	99.97%	100%	100%
N	99.47%	99.74%	77.19%	83.96%	77.19%	79.25%
F	97.38%	76.67%	77.19%	79.20%	77.19%	79.25%
%Age average	98.38%	94.07%	90.08%	81.24%	91%	80.30%

**Table 9:** Comparison result of proposed CAA-TL model with literature.

Studies	Data augmentation	Dataset used	Method		Findings

Strodthoff et al. [2]	No	PTB -XL	ResNet and inception		-Predicted accuracy 89.8% -Less accurate

Wasimuddin et al. [5]	No	ECG-ID	CAD and machine learning		-Predicted accuracy 98.5% -Handcrafted

Vijayakumar et al. [6]	No	No	Feature extraction to remove noise		-Predicted accuracy 94.5% -Handcrafted

Hsu et al. [14]	No	MIT-DB	AlexNet and ResNet		-Predicted accuracy 94.4% -Fewer images

Acharya et al. [16]	No	PTB DB	CNN layers		-Accuracy 93.5% with noise and 95.22% without noise Less accurate

Gaddam et al. [37]	No	MIT-DB	AlexNet		-Predicted accuracy 95.6% -Only 1 approach was used with less accuracy

Reddy and khare [32]	No	UCI dataset	Rule-based fuzzy classifier and feature reduction		-Predicted accuracy 76.51% -Handcrafted

Poudel et al. [34]	No	KVASIR dataset	CAD and machine learning		F1-score of 0.88 -Handcrafted

Siddique et al. [36]	No	Private	Fuzzy inference system, deep extreme machine learning, and ANN		87.05%, 92.45%, and 89.4% -Handcrafted

Proposed CAA-TL model	Yes	MIT-BIH	Transfer LearningMethods	AlexNet	Accuracy (98.38%)
				SqueezeNet	Accuracy (90.08%)
				ResNet50	Accuracy (91%)

The article "ECG Classification for Detecting ECG Arrhythmia Empowered with Deep Learning Approaches" was published in 2022. Journal: Comput Intell Neurosci.

## Data Availability

The data used in this paper can be requested from the corresponding author upon request.
